RETRACTED

# High bioavailablilty iron maize (*Zea mays* L.) developed through molecular breeding provides more absorbable iron in vitro (*Caco-2* model) and in vivo (*Gallus gallus*)

**DOI:** 10.1186/1475-2891-12-3

**Published:** 2013-01-04

**Authors:** Elad Tako, Owen A Hoekenga, Leon V Kochian, Raymond P Glahn

**Affiliations:** 1 USDA-ARS Robert W. Holley Center for Agriculture and Health, 538 Tower Road, Cornell University, Ithaca, NY, 14853, USA

**Keywords:** Maize, Biofortification, Iron bioavailability, In vitro digestion/Caco- 2 cell model, Broiler chicken, Intestine

## Abstract

**Background:**

Iron (Fe) deficiency is the most common micronutrient deficiency worldwide. Iron biofortification is a preventative strategy that alleviates Fe deficiency by improving the amount of absorbable Fe in crops. In the present study, we used an in vitro digestion/Caco 2 cell culture model as the guiding tool for breeding and development of two maize (*Zea mays* L.) lines with contrasting Fe bioavailability (ie. Low and High). Our objective was to confirm and validate the in vitro results and approach. Also, to compare the capacities of our two maize hybrid varieties to deliver Fe for hemoglobin (Hb) synthesis and to improve the Fe status of Fe deficient broiler chickens.

**Methods:**

We compared the Fe-bioavailability between these two maize varieties with the presence or absence of added Fe in the maize based-diets. Diets were made with 75% (w/w) maize of either low or high Fe-bioavailability maize, with or without Fe (ferric citrate). Chicks (*Gallus gallus*) were fed the diets for 6 wk. Hb, liver ferritin and Fe related transporter/enzyme gene-expression were measured. Hemoglobin maintenance efficiency (HME) and total body Hb Fe values were used to estimate Fe bioavailability from the diets.

**Results:**

DMT-1, DcytB and ferroportin expressions were higher (P < 0.05) in the "Low Fe" group than in the "High Fe" group (no added Fe), indicating lower Fe status and adaptation to less Fe-bioavailability. At times, Hb concentrations (d 21,28,35), HME (d 21), Hb-Fe (as from d 14) and liver ferritin were higher in the "High Fe" than in the "Low Fe" groups (P < 0.05), indicating greater Fe absorption from the diet and improved Fe status.

**Conclusions:**

We conclude that the High Fe-bioavailability maize contains more bioavailable Fe than the Low Fe-bioavailability maize, presumably due to a more favorable matrix for absorption. Maize shows promise for Fe biofortification; therefore, human trials should be conducted to determine the efficacy of consuming the high bioavailable Fe maize to reduce Fe deficiency.

## Introduction

Iron (Fe) deficiency affects one-third of the world's population [1]. Iron is vital for oxygen transport and energy metabolism [2]. The consequences of Fe deficiency anemia include impaired growth, retarded psychomotor and cognitive development, damaged immune mechanisms with increased morbidity and mortality rates [1,3].

RETRACTED

Efforts to decrease dietary Fe deficiency utilize fortification, supplementation and diversification of diets. These strategies had limited success in resource-limited environments and poor countries due to cost, limited health care, and availability of food processing facilities [4-7]. Hence, genetic improvement (biofortification) of staple crops is an attractive alternative to dietary fortification or diversification, as delivery of the Fe-rich staple is achieved through the development and promotion of new plant varieties that are aimed to alleviate dietary Fe deficiency and anemia [7].

Maize (*Zea mays* L.) is widely consumed in developing countries and provides energy, vitamins and minerals [8-15]. However, a major cause of Fe deficiency is poor intake of Fe, due to low bioavailability from plant-based diets containing mineral absorption inhibitors as polyphenols and phytates. In the most maize-dependent countries, where maize provides ≥ 20% of dietary protein, Fe deficiency and anemia are prevalent [1,16-18]. Hence, maize is an attractive candidate for Fe biofortification.

Increased Fe concentration in staple food crops may not necessarily translate into a proportional increase in absorbed Fe, because crop varieties with high Fe concentrations may have increased (or decreased) concentrations of Fe absorption inhibitors or enhancers. It is necessary to measure the amount of Fe concentration and bioavailability in new Fe-enhanced crops. The in vitro screening employs a simulated gastric and intestinal digestion of food coupled with culture of human intestinal cells [19]. This bioassay is necessary to pinpoint genetic markers for Fe bioavailability.

Research into the genetic basis for Fe nutritional quality in maize has established the potential for Fe biofortification, as Fe concentration and bioavailability are under genetic control and have demonstrated potential for improvement [8,9]. Previously, we utilized quantitative trait locus (QTL) mapping to characterize the genetic complexity of Fe concentration and bioavailability in maize [9,20,21]. New varieties were developed using members of the mapping population, that were largely identical except in the chromosomal regions surrounding the 3 QTL with largest effect on Fe bioavailability. These derivatives were selected to create a maximal degree of contrast in predicted Fe bioavailability. With High and Low varieties in both parental backgrounds, these High-Fe and Low-Fe bioavailability hybrids are essentially identical for all parts of their genomes (all features of grain quality would be expected to be the same) except the 3 QTL-containing regions on maize chromosomes 3, 6 and 9 [8,9]. Preliminary in vivo study indicated that the predictions made with the Caco-2 bioassay were valid for predicting Fe bioavailability [8]. The equivalence of the High-Fe and Low-Fe bioavailability varieties for grain Fe concentration, flowering time, and other characteristics except Fe bioavailability suggests that our strategy of creating these hybrids and the focus on the effect of the 3 major QTL was successful [8,9].

RETRACTED

The poultry model have been used for nutritional research and was shown to be an excellent animal to model Fe bioavailability, as chicks respond quickly to malnutrition, and their micronutrient deficient phenotypes include poor Fe status, growth stunting, and organ hypertrophy [22-24]. Also, this model agrees well with human cell line in vitro results [22-25]. Hence, the objective of the current study was to compare the capacities of our two new maize hybrid varieties to deliver Fe for hemoglobin synthesis and to improve the Fe status of Fe deficient broiler chickens.

## Materials and methods

### Creation of high-Fe bioavailability and low-Fe bioavailability maize varieties

QTL-mapping is the process of utilizing genetically mapped varieties coupled with a biological measurement (as Fe bioavailability) and then utilizing statistics to correlate that measurement with genetic markers. QTL-mapping revealed that Fe concentration in maize grain was under the control of at least 10 regulatory factors on 6 of the 10 chromosomes of maize [9]. However, Fe-bioavailability was regulated by fewer, larger QTL, which suggested that this trait might be easier to manipulate. Furthermore, Fe concentration and bioavailability had only a small positive association between them indicating that Fe concentration differences between members of the mapping population were not driving the differences in Fe bioavailability [9]. Derivation of the High-Fe and Low-Fe bioavailability maize hybrids was previously described [8,9]. Briefly, The Caco-2 bioassay was the guiding tool for the measure of Fe bioavailability in the maize grain [9]. Statistical analysis was used to identify molecular markers (i.e. QTL) associated with Fe bioavailability. These markers were used to select sister lines that contrasted for the 3 largest effect QTL in order to create new varieties that were highly genetically similar but different (high or low) for Fe-bioavailability. As sister lines were created in both of the parental genetic backgrounds used in the mapping population, nearly isogenic hybrids were made by crossing the parents lines (*high* with *high* and *low* with *low*). These hybrids were heterozygous everywhere except the 3 Fe-bioavailability QTL [9] and were similar except for bioavailable-Fe in the whole grain [8] (Figure 1). The High-Fe and Low-Fe maize were produced using standard agronomic practices at the Cornell University Research Farm (Poplar Ridge, NY) in the summer of 2009. Plots were mechanically planted and harvested. Grain was dried to ~12% moisture, processed in bulk (~ 800 Kg of each variety), and stored at 4°C until the feeding study began. In preparation for the in vivo trial, maize grains were thoroughly washed in _dd_H2O prior to cooking and freeze drying. Maize varieties were ground prior to mixing the diets.

RETRACTED

**Figure 1:** **Description of maize (*Zea mays *L.) varieties used in this study.**

### Animals, diets and study design

One hundred and twenty fertile Cornish cross broiler eggs were obtained from a commercial hatchery (Moyer’s Chicks, Quakertown, PA). Eggs were incubated under optimal conditions at the Cornell University Animal Science poultry farm incubator. Upon hatching (92% hatchability), chicks were allocated into 4 treatment groups on the basis of body weight, gender and blood hemoglobin concentration (aimed to ensure equal distribution between groups, n=10): 1. "High + Fe": 75% High-Fe bioavailability cooked maize with added Fe based diet (65 μg/g Fe). 2. "High": 75% High-Fe bioavailability cooked maize with no Fe added based diet (24 μg/g Fe). 3. "Low + Fe": 75% Low-Fe bioavailability cooked maize with added Fe based diet (66 μg/g Fe). 4. "Low": 75% Low-Fe bioavailability cooked maize with no Fe added based diet (23 μg/g Fe) (Table 1). Cooked/raw maize were compared as in vitro pilot studies indicated that cooking may increase the difference in Fe bioavailability between the two lines. Chicks were housed in a total-confinement building (1 chick per 0.5 m^2^ cage). Birds were under indoor controlled temperatures and were provided 16 h of light. Cages were equipped with an automatic nipple drinker and manual self feeder. All birds were given *ad libitum* access to water (Fe concentration was 0.379±0.012 μg/g). Iron concentrations in the water and diets were determined by an inductively-coupled argon-plasma/atomic emission spectrophotometer (ICAP 61E Thermal Jarrell Ash Trace Analyzer, Jarrell Ash Co. Franklin, MA) following wet ashing. Feed intakes were measured daily (from day 1). Iron intakes were calculated from feed intakes and Fe concentration in the diets.

**Table 1:** Composition of experimental diets

**Ingredient**	**"High+Fe" Diet**	**"High" Diet**	**"Low+Fe" Diet**	**"Low" Diet**
***g/Kg*diet (by formulation)**				
High-Fe bioavailability Maize (21 μg Fe/g)	750	750	-	-
Low-Fe bioavailability Maize (20 μg Fe/g)	-	-	750	750
Dry skim milk	100	100	100	100
DL-Methionine	2.5	2.5	2.5	2.5
Corn oil	30	30	30	30
Corn starch	46.50	46.75	46.50	46.75
Choline Chloride	0.75	0.75	0.75	0.75
Vit/Min^1^ (no Fe)	70	70	70	70
Ferric citrate	0.25	-	0.25	-
Total	1000	1000	1000	1000
Concentrations of selected components means±SEM, n=10 (by analysis)^4^				
Fe, *μgFe/g* diet^2^	65.3±0.9^a^	24.5±1.0^b^	66.1±2.4^a^	23.6±0.2^b^
Phytate, *μmol/g* diet^3^	10.2 ± 0.2^a^	10.1 ±0.2^a^	10.1 ± 0.2^a^	10.0 ±0.2^a^

^1^Vitamin and mineral premix provided/kg diet (330002 Chick vitamin mixture; 230000 Salt mix for chick diet; *Dyets* Inc. Bethlehem, PA).

^2^Dietary iron concentrations analysis is described in the materials and methods section.

^3^Method for determining phytate contents are described in the materials and methods section.

^4^Values are means±SEM. ^a,b^Within a row, means without a common letter are significantly different, P < 0.05.

RETRACTED

### Blood analysis and hemoglobin (Hb) measurements

Blood samples were collected from the wing vein (n=10,~100 μL) using micro-hematocrit heparinized capillary tubes^a^ (Fisher, Pittsburgh, PA). Samples were collected following an 8 h overnight feed deprivation. Samples were analyzed for Hb concentration (see below). Body weights (BW) and Hb concentrations were measured weekly.

Fe-bioavailability was calculated as hemoglobin maintenance efficiency (HME) [23-29]:

(1) $$\mathrm{HME}=\frac{\mathrm{Hb}\;\mathrm{Fe},\;\mathrm{mg}\;\left(\mathrm{final}\right)-\mathrm{Hb}\;\mathrm{Fe},\;\mathrm{mg}\;\left(\mathrm{initial}\right)}{\mathrm{Total}\;\mathrm{Fe}\;\mathrm{Intake},\;\mathrm{mg}}\;\times \;100$$

Where Hb-Fe (index of Fe absorption) = total body hemoglobin Fe. Hb-Fe was calculated from hemoglobin concentrations and estimates of blood volume based on BW (a blood volume of 85 mL per kg body weight is assumed) [23-25,28]:

(2) $$\mathrm{Hb}-\mathrm{Fe}\;\left(\mathrm{mg}\right)=\mathrm{BW}\;\left(\mathrm{kg}\right)\times 0.085\;L\;\mathrm{blood}/\mathrm{kg}\times \mathrm{Hb}\;\left(g/L\right)\times 3.35\mathrm{mg}\;\mathrm{Fe}/g\;\mathrm{Hb}.$$

Fe intakes were calculated from feed intake data and Fe concentrations in the feed.

Blood Hb concentrations were determined spectrophotometrically using the cyanmethemoglobin method (H7506-STD, Pointe Scientific Inc. Canton, MI) following the kit manufacturer’s instructions.

At the end of the experiment (day 42), birds were euthanized by carbon-dioxide exposure. The digestive tracts and livers were quickly removed and separated. Tissue samples were taken from the small intestine and liver (~ 1–2 cm; ~2-3 g, respectively). The samples were immediately frozen in liquid nitrogen, and then stored in a -80°C freezer until analysis.

RETRACTED

All animal protocols were approved by the Cornell University Institutional Animal Care and Use Committee.

### Isolation of total RNA

Total RNA was extracted from 30 mg of the proximal duodenal tissue (n=10) using Qiagen RNeasy Mini Kit (RNeasy Mini Kit, Qiagen Inc.,Valencia, CA) according to the manufacturer’s protocol. Total RNA was eluted in 50 μL of RNase free water. All steps were carried out under RNase free conditions. RNA was quantified by absorbance at *A*_*260/280*_. Integrity of the 28S and 18S ribosomal RNAs was verified by 1.5% agarose gel electrophoresis followed by ethidium-bromide staining. DNA contamination was removed using TURBO DNase treatment and removal kit from AMBION (Austin, TX, USA).

### DMT1, DcytB and ferroprtin gene expression analysis

As previously described [23-25,27,30], Divalent metal transporter-1 (DMT1); Duodenal cytochrome-B **(**DcytB) and Ferroprtin mRNA levels in duodenal mucosa were analyzed by quantitative real-time RT-PCR (20 μL reactions); values were normalized to 18S expression. The total RNA was reverse-transcribed to complementary DNA in a 25 μL volume containing 1 μg of extracted RNA. Reverse-transcription was carried out using the Superscript-First Strand Synthesis Kit for reverse-transcription PCR according to the manufacturer’s protocol (Invitrogen, Carlsbad, CA). Gene-specific primers were designed using Primer Express software (Applied Biosystems, Carlsbad, CA) chosen from the fragment of the chicken (*Gallus gallus*) duodenal *DMT1* gene (GeneBank database; GI 206597489) (forward: 5’-AGC CGT TCA CCA CTT ATT TCG-3’; reverse: 5’-GGT CCA AAT AGG CGA TGC TC-3’), *DcytB* gene (GI 20380692) (forward: 5’-GGC CGT GTT TGA GAA CCA CAA TGT T-3’; reverse: 5’-CGT TTG CAA TCA CGT TTC CAA AGA T-3’) and *Ferroportin* gene (GI 61098365) (forward: 5’-GAT GCA TTC TGA ACA ACC AAG GA’; reverse: 5’-GGA GAC TGG GTG GAC AAG AAC TC-3’). *Ribosomal 18S* was used to normalize the results (GI 7262899) (forward: 5’- CGA TGC TCT TAA CTG AGT-3’; reverse: 5’-CAG CTT TGC AAC CAT ACT C-3’). Real-time PCR was performed in a 7500 Real-Time PCR system instrument (Applied Biosystem, Carlsbad, CA). The 20 μL PCR mixture consisted of 10 μL of POWER SYBR Green PCR Master Mix (Applied Biosystem, Carlsbad, CA), 5 μL of water, and 1 μL of each primer that was added to 3 μL of the cDNA diluted 1:25. All reactions were performed in duplicates and under the following conditions: 50°C for 2 min, 95°C for 2 min, 42 cycles of 95°C for 30 s, and 60°C for 1 min. Also, to ensure amplification of a single product, a dissociation curve was determined under the following conditions: 95°C for 1 min, 55°C for 30 s, and 95°C for 30 s. Specificity of the product was also confirmed by running samples on a 1.5% agarose gel, excising for purification using the QIAquick Gel Extraction Kit (QIAGEN, Valencia, CA). Calculations of threshold cycles, amplification efficiencies, and *R*0 values (the starting fluorescence value that is proportional to the relative starting template concentration) were performed using the data analysis for real-time PCR *Excel* workbook and as previously described [31].

RETRACTED

### Ferritin and Fe in the liver

We followed previously described procedures [23,24,32,33]. Briefly, 1 g of sample was diluted into 1 mL of 50 mM Hepes buffer, pH 7.4, and homogenized on ice for 2 min (5000 g). One mL of each homogenate was subjected to heat treatment for 10 min at 75°C to aid isolation of ferritin (other proteins are not stable at that temperature). Subsequently, samples were immediately cooled down on ice for 30 min. Thereafter, samples were centrifuged for 30 min (13000 g) at 4°C until a clear supernatant was obtained and the pellet containing most of the insoluble denaturated proteins was discarded. Iron concentrations in the liver samples were determined by an inductively-coupled argon-plasma/atomic emission spectrophotometer (ICAP 61E Thermal Jarrell Ash Trace Analyzer, Jarrell Ash Co. Franklin, MA) following wet ashing.

### Electrophoresis, staining and measurement of gels

Native polyacrylamide gel electrophoresis was conducted using a 6% separating gel and a 5% stacking gel. Samples were run at a constant voltage of 100 V. Thereafter, gels were treated with either of the two stains: Coomasie blue G-250 stain, specific for proteins, or potassium ferricyanide (K_3_Fe(CN)_6_) stain, specific for Fe. The corresponding band found in the protein and Fe stained gel was considered to be ferritin [23,24,32,33].

Measurements of the bands were conducted using the Quantity-One-1-D analysis program (Bio-Rad, Hercules, CA). The local background was subtracted from each sample. Horse spleen ferritin (Sigma Aldrich Co., St. Louis, MO) was used as a standard for calibrating ferritin protein and Fe concentrations of the samples. Dilutions of the horse spleen ferritin were made and treated similarly to the liver supernatant samples in order to create a reference line for both protein and Fe-stained gels [23,24,32,33].

### In-vitro iron bioavailability assessment

An in vitro digestion/Caco-2 cell culture model [19,23-28,34,35] was used to assess Fe-bioavailability. The maize only samples (High- Fe bioavailability maize; Low-Fe bioavailability maize and control-commercial maize) and the diets (High diet; Low diet; High + Fe diet; Low + Fe diet) were subjected to simulated gastric and intestinal digestion. Briefly, the intestinal digestion is carried out in cylindrical inserts closed on the bottom by a semipermeable membrane and placed in wells containing Caco-2 cell monolayers bathed in culture medium. The upper chamber was formed by fitting the bottom of Transwell insert ring (Corning) with a 15000 Da molecular weight cut off (MWCO) membrane (Spectra/Por 2.1, Spectrum Medical, Gardena, CA). The dialysis membrane was held in place using a silicone ring (Web Seal, Rochester, NY).

RETRACTED

Iron uptake by the Caco-2 cell monolayers was assessed by measuring *ferritin* concentrations in the cells. Six replicates of each Fe bioavailability measurement were performed. In terms of materials for the study, Caco-2 cells were obtained from the American Type Culture Collection (Rockville, MD) at passage 17 and used in experiments at passage 29. Cells were seeded at densities of 50,000 cells/cm^2^ in collagen-treated 6 well plates (Costar Corp., Cambridge, MA). The integrity of the monolayer was verified by optical microscopy. The cells were cultured at 37°C in an incubator with 5% CO_2_ and 95% air atmosphere at constant humidity, and the medium was changed every 48 h.

The cells were maintained in Dulbecco’s modified Eagle medium plus 1% antibiotic/antimycotic solution, 25 mmol/L HEPES, and 10% fetal bovine serum. 48 h prior the experiment, the growth medium was removed from culture wells, the cell layer was washed, and the growth medium was replaced with minimum essential media (MEM) at pH 7.0. The MEM was supplemented with 10 mmol/L PIPES, 1% antibiotic/antimycotic solution, 4 mg/L hydrocortisone, 5 mg/L insulin, 5 μg/L selenium, 34 μg/L triiodothyronine, and 20 μg/L epidermal growth factor. This enriched MEM contained less than 80 μg Fe/L.

All ingredients and supplements for cell culture media were obtained from GIBCO (Rockville, MD). The cells were used in the Fe uptake experiment at 13 days post seeding. In these conditions, the amount of cell protein measured in each well was highly consistent between wells. On experiment day, 1.5 mL of the digested sample was added to the insert’s upper chamber and incubated for 2 h. Then, inserts were removed and 1 mL of MEM was added. Cell cultures were incubated for 22 h at 37°C.

It was previously shown that intracellular ascorbic acid status might influence ferritin formation (i.e. cellular Fe uptake), and Fe related transporters and enzyme expression in Caco-2 cells [23,24,34]. In the current study, samples were not added with ascorbic acid when Fe bioavailability was tested in vitro.

RETRACTED

### Harvesting of caco-2 cells for ferritin analysis

The ferritin and total protein contents analyses protocols were previously described [19,23,24,35]. Briefly, growth medium was removed from the culture well by aspiration and the cells were washed twice with a solution containing 140 mmol/L NaCl, 5 mmol/L KCl, and 10 mmol/L PIPES at pH 7.0. The cells were harvested by adding an aliquot of deionized water and placing them in a sonicator (Lab-Line instruments, Melrose Park, IL).

The ferritin and total protein concentrations were determined on an aliquot of the harvested cell suspension with a one-stage sandwich immunoradiometric assay (FER-IRON II Ferritin assay, Ramco laboratories, Houston, TX) and a colorimetric assay (Bio-Rad DC Protein assay, Bio-Rad, Hercules, CA), respectively. Caco-2 cells synthesize ferritin in response to increases in intracellular Fe concentration. Therefore, we used the ratio of ferritin/total protein (expressed as ng ferritin/mg protein) as an index of the cellular Fe-uptake.

### Phytate content in diets

A Dionex liquid (Dionex Corp. Sunnyvale, CA) chromatograph system (AS50 autosampler), equipped with conductivity detector model ED50, and gradient pump GS50 were used along with an IonPac AG11 guard column and IonPac AS11 column (4×250 mm) to quantify phytate. PeakNet 6.40 software was used to process chromatographic data. The mobile phases were (A) 200 mmol/L NaOH (carbonate-free) and (B) deionized water, using a flow rate of 1 mL/min. Phytate was extracted from 250 mg of dry, lyophilized diet sample, in 10mL of a 1.25% H_2_SO4 solution; the extraction process was 2 h, after which the samples were centrifuged at 3660 *g* for 10 min. Subsamples were diluted 1:10 with deionized water, and 10 *μ*L was injected and analyzed (n=10).

### Statistical analyses

Results were analyzed by ANOVA using the general linear models procedure of SAS software (SAS Institute Inc. Cary, NC). Differences between treatments were compared by Tukey’s test were considered statisticant at P < 0.050. Values in the text are means ± SEM.

## Results

### Hemoglobin (Hb), Hb Fe and Hb maintenance efficiency (HME)

No significant differences were measured in body weights between treatment groups (P > 0.05). However, as from day 21 of the study, hemoglobin (Hb) concentrations were higher (P < 0.05) in the "High" group than in the "Low" group. In addition, as from day 14, Hb-Fe values were higher in the "High" group than in the "Low" group; the increase in total body Hb-Fe from the beginning of the study to the end of the 6th wk was significantly greater in the "High" group than in the "Low" group (12.8 ± 0.5 mg vs. 9.7 ± 0.3 mg, respectively, P < 0.05, Table 2). Significant differences in HME (P < 0.05) were measured between the "High" group and "Low" group on day 21 (P < 0.05). Also, significant differences in HME (P < 0.05) were measured between the "High + Fe" and "Low + Fe" groups on days 28 and 42 (P < 0.05, Table 2).

RETRACTED

**Table 2:** **Hemoglobin (Hb, g/L), Total body Hb-Fe content (mg) and hemoglobin maintenance efficiency**^**1**^**(HME, %) in chicken fed the tested diets from d 0 to d 42**^**2**^

**Treatment**^**3**^		**Day 0**	**Day 7**	**Day 14**	**Day 21**	**Day 28**	**Day 35**	**Day 42**
"High + Fe"	Hb	92^a^±9.0	88^a^±5.0	104^a^ ±11	102^a^ ±6.0	102^a^ ±5.0	97^a^ ±13	97^a^ ±7.0
	Hb Fe	1.02^a^ ±0.1	2.52^a^±0.2	4.35^a^ ±0.4	5.80^a^ ±0.4	8.35^a^ ±0.6	9.62^a^ ±0.6	16.49^a^ ±0.7
	HME	-	22.7^b^ ±2.9	22.5^bc^ ±2.9	19.8^bc^±2.5	20.1^b^ ±2.6	15.8^b^ ±2.0	20.2^b^ ±2.6
"Low + Fe"	Hb	92^a^±9.0	86^a^±8.0	100^a^ ±13	94^ab^ ±14	94^ab^ ±6.0	88^a^ ±6.0	87^a^ ±3.0
	Hb Fe	1.02^a^ ±0.1	2.30^a^±0.2	4.28^a^ ±0.3	5.53^a^ ±0.4	7.72^a^ ±0.5	8.84^ab^±0.6	14.52^ab^±0.7
	HME	-	18.5^b^ ±2.4	19.2^c^±2.5	15.4^c^ ±2.0	14.4^c^ ±1.9	11.3^bc^±1.5	13.8^c^ ±1.7
"High"	Hb	92^a^±9.0	88^a^±6.0	76^b^ ±3.0	81^b^ ±3.0	81^b^ ±4.0	82^a^ ±7.0	82^ab^ ±9.0
	Hb Fe	1.02^a^ ±0.1	2.37^a^±0.1	3.04^b^ ±0.2	4.72^b^ ±0.2	6.30^b^ ±0.4	8.07^b^ ±0.5	13.79^b^ ±1.0
	HME	-	58.4^a^ ±7.6	37.8^a^ ±4.9	40.3^a^ ±5.2	37.7^a^ ±4.9	35.3^a^ ±4.6	44.9^a^ ±5.8
"Low"	Hb	92^a^±9.0	82^a^±5.0	70^b^ ±3.0	66^c^ ±7.0	66^c^ ±5.0	68^b^ ±4.0	67^b^ ±8.0
	Hb Fe	1.02^a^ ±0.1	2.21^a^±0.1	2.54^c^ ±0.2	3.41^c^ ±0.2	4.62^c^ ±0.3	6.29^c^ ±0.4	10.73^c^ ±0.6
	HME	-	52.1^a^ ±6.7	29.7^ab^±3.8	28.0^b^ ±3.6	27.1^ab^ ±3.5	27.7^a^ ±3.6	35.8^a^ ±4.6

^a,b,c^Within a column and for each parameter (i.e. Hb, Hb Fe, HME), treatment group means without a common letter differ, P < 0.05.

^1^Calculations are described in the materials and methods section.

^2^Values are means±SEM, n=10.

^3^The experimental diets are described in the materials and methods section.

### Ferritin and iron in the liver

Avian ferritins corresponded to a weight of approximately 470 to 500 kDa [23,24,32,33,36]. Liver Fe and ferritin concentrations were higher in the "High" group than in the "Low" group (n=10, P < 0.05, Table 3).

**Table 3:** **Liver ferritin protein and liver iron**^**1**^**concentration in chicken given the treatment diets**

**Treatment**	**Liver ferritin**^**1**^**,*μg/g*wet weight**	**Liver iron**^**2**^**,*μg/g*tissue**
"High + Fe"	650±18^a^	64.3±3.8^a^
"Low + Fe"	645±22^a^	39.6±2.3^c^
"High"	435±13^b^	52.2±3.1^b^
"Low"	355±10^c^	43.3±2.5^c^

^a,b,c^Within a column and for each parameter (i.e. liver ferritin or liver Fe), treatment group means without a common letter differ, P< 0.05 (values are mean±SEM, n=10).

^1^Atomic mass for iron is 55.8 *g/mol*.

^2^Liver tissue iron concentrations analysis is described in the materials and methods section.

RETRACTED

### Gene expression of iron transporters (DMT-1, Ferroportin) and iron reductase (DcytB) in the duodenum

Gene expression analysis of duodenal DMT-1, Ferroportin and DcytB, with results reported relative to 18S rRNA, revealed greater mRNA levels for DMT1, DcytB and Ferroportin in the "Low" group compared to the "High" group (mean±SEM) (n=10, P < 0.05, Figure 2).

**Figure 2:** **Duodenum mRNA expression of DMT1, divalent metal transporter 1; DcytB, duodenal cytochrome b reductase; and ferroportin in chickens at the age 6 weeks.** Changes in mRNA expression are shown relative to expression of 18S rRNA in arbitrary units (AU). Values are means ± SEM, n = 10, P < 0.05.

### Caco-2 cell ferritin protein formation

An in vitro digestion/Caco-2 cell culture model was used to evaluate Fe bioavailability from the tested maize only and maize based diets by measuring ferritin formation in the cells (ie. a measure of cell Fe uptake) following exposure to digests of the samples. The amount of bioavailable iron in vitro was significantly higher (P < 0.05) in the "High" and "High + Fe" diets than in the "Low" and "Low + Fe" diets (mean±SEM) (n=6, P < 0.05, Table 4).

**Table 4:** **Ferritin concentrations in Caco-2 cells exposed to samples of maize only and maize-based diet digests; and Fe concentrations in samples of maize only and maize-based diet digests**^**1**^

**Tested sample**	**Caco-2 Cell Ferritin**^**2**^**, ng/mg of total protein**	**Fe concentration**^**3**^**, μg/g sample**
High Fe maize only	22.51±0.9^c^	20.9 ±0.2^c^
Low Fe maize only	13.40 ±0.6^d^	20.0 ±0.9^c^
"High + Fe" diet	74.36 ±1.6^a^	65.3 ±0.9^a^
"Low + Fe" diet	56.89 ±1.1^b^	66.1 ±2.4^a^
"High" diet	6.55 ±0.5^e^	24.5 ±1.0^b^
"Low" Diet	1.31 ±0.4^f^	23.6 ±0.2^bc^

^1^Values are means ± SEM, n = 6.

^a,b,c,d,e,f^ Within a column (ferritin or Fe concentrations), means without a common letter differ, P < 0.05.

^2^Caco-2 bioassay procedures and preparation of the digested samples are described in the materials and methods section.

^3^Dietary iron concentrations analysis is described in the materials and methods section.

### Phytate concentration in the diet samples

No significant differences in phytate concentration (IP_6_) were measured between treatments diets (n=5; P > 0.05, Table 1).

## Discussion

Maize is an important component of the human food supply, especially in Eastern and Southern Africa, the Caribbean, and the Andean region of South America [1]. In these regions where dietary Fe deficiency and anemia are common and are a critical health concern, maize is often a component of every meal [1,37-40]. Hence, increasing Fe bioavailability in maize has potential to alleviate dietary Fe deficiency.

RETRACTED

Biofortification is the process of enriching the nutrient quality of staple food crops via plant breeding [38,40], as a nutritional agricultural intervention it can provide a sustainable source of micronutrients to at risk populations [41]. Iron biofortifcation and bioavailability from plant foods is influenced by many factors, especially polyphenols and phytic acid [42]. Iron biofortification can be done via enhancement of concentration and or bioavailability, and recent studies indicate that both factors have a genetic basis but are also greatly influenced by environment and genotype by environment interactions [43,44]. Given the generally low Fe bioavailability in staple crops, enhancing the bioavailable fraction of Fe rather than merely increasing the total concentration may represent an improved path for Fe biofortification [8,9,44,45]. Additionally, the correlation between bioavailable-Fe and total-Fe is not always robust while both traits may have similar genetic complexity [9].

Crop improvement via conventional breeding can produce vast numbers of varieties [46]. Only a fraction of these genetically distinct individuals will have the desired gain in quality to justify being released as a new variety. The selection process is a key issue. One option could be the target of selection in order to biofortify maize. Hence, Fe concentration is an obvious choice, as its evaluation is amenable to high-throughput screening methods [47]. For maize and wheat, Fe concentration is not well correlated with Fe bioavailability, while these traits are correlated in beans [9,23,24].

The mechanisms that modulate Fe bioavailability are unclear, therefore, estimating Fe bioavailability is important. We employed the Caco-2 bioassay as part of a recursive process to create maize varieties with different levels of bioavailable-Fe [9,19,23-28,48,49]. The bioassay was used to evaluate 145 members of a maize mapping population, where neither Fe concentration nor phytate levels were well correlated with bioavailable-Fe [9]. Also, molecular genetic markers were used to evaluate nearly 700 genetically distinct individuals from our breeding program in order to create the 4 varieties that were selected to differ in bioavailable-Fe. Molecular breeding approaches with these 4 inbred varieties were used to create the 2 hybrids evaluated in this study and our preliminary study [8].

The observation that bioavailable-Fe was being modulated through the course of our breeding strategy needed verification beyond the Caco-2 bioassay. This assay also indicated that Fe bioavailability could be reliably modified across several years in NY and other sites in North America [9]. The current results demonstrate that Caco-2/QTL approach can be used to enhance maize Fe bioavailability. Also, if adequate mapping populations are available, this approach can be extended to other crops.

RETRACTED

In this study the maize lines were grown under standard agronomic conditions on a research farm, similar to other varieties of maize grown that summer. This demonstrates that the High and Low Fe bioavailability varieties can be grown using production scale agriculture. Current study followed a previous study, where similar results were obtained with smaller amounts of maize (~30 kg), where all plants were hand pollinated and harvested [8]. Thus we have demonstrated that the nutritional differential between the High and Low Fe bioavailability varieties can be created and maintained in consecutive years using different field practices. This benefit was confirmed as birds receiving the High-Fe bioavailability maize diets had improved Fe status as their liver Fe and ferritin concentrations (Table 3), and body Hb-Fe (Table 2) were higher (P < 0.05) than birds receiving the Low-Fe bioavailability maize diets. The low-Fe bioavailability maize-fed birds had elevated expression of DMT1, DcytB and Ferroportin, which indicates adaptation to the low Fe bioavailability (Figure 2).

Iron biofortification of crops can be accomplished via an increase in concentration or an increase in bioavailability. Either way, the net result is that more Fe is delivered for absorption. Increased Fe concentrations in beans [24,26] and rice [38,50] have a beneficial effect on the Fe status in vivo; in a human study [50] Fe-biofortified rice improved Fe stores in Fe-deficient (not anemic) women, even though Fe concentrations in the rice were low (3.2 μg/g and 0.57 μg/g for the high Fe and control rice, respectively). Recently, the effects of high-Fe (71 μg/g) and standard-Fe (49 μg/g) red mottled Andean beans, on Fe status of chickens were investigated. Final body Hb-Fe contents were different between the standard (12.58±1.0 mg) and high Fe (15.04 ± 0.65 mg) bean groups (P < 0.05). DMT-1, DcytB and ferroportin expression were higher and liver ferritin was lower (P < 0.05) in the standard group vs. the biofortified group, indicating a physiological effort to compensate for lower dietary-Fe. In vitro analysis showed lower Fe bioavailability in cells exposed to standard bean based diet. It was concluded that the higher Fe beans provided more bioavailable-Fe than standard beans [24]. These studies showed that the higher Fe concentration improved Fe status, as no difference in percent bioavailability was apparent. However, in the present study, Fe concentration was similar yet the amount that was bioavailable from the High-Fe bioavailability maize was higher.

RETRACTED

Many cereal grains as maize are rich with phytate that may decrease mineral bioavailability [8,9,51-53]. Our study suggests that it is possible to counteract the Fe absorption inhibitory effect of phytate and possibly other inhibitors by increasing Fe bioavailability (not necessarily concentration). This knowledge is vital for developing plant breeding strategies as part of the continuing battle with dietary Fe deficiency.

Iron deficiency is a worldwide, endemic public health problem. Food system-based interventions such as biofortification are a practical and sustainable solution for at risk populations [7]. An efficacy trial comparing biofortified and standard maize in human populations is now warranted.

## Conclusions

Based on the data shown here, we conclude that the enhanced bioavailable-Fe maize we have generated via a molecular plant breeding strategy is a promising vehicle for alleviating Fe deficiency in human populations where maize is a major dietary staple.

The results presented in this study show that breeding can improve the Fe quality in maize. These findings demonstrate the potential for Fe biofortification in maize.

## Endnote

^a^Mention of a trademark, proprietary product or vendor does not constitute a guarantee or warranty of the product by the United states Department of Agriculture and does not imply its approval to the exclusion of other products or vendors that may also be suitable.

## Abbreviations

Fe: Iron; Hb: Hemoglobin; Hb-Fe: Hemoglobin-Iron; HME: Hemoglobin maintenance efficiency; DMT-1: Divalent metal transporter 1; DcytB: Duodenal cytochrome B; QTL: Quantitative trait locus.

## Competing interests

The authors declare no conflict of interest.

## Authors’ contributions

ET designed research, conducted research, collected and analyzed data and wrote the paper. OAH designed research, created and provided the High Fe and Low Fe maize varieties, and co-authored the paper. LVK co-authored the paper. RPG designed research, and co-authored the paper. All authors read and approved the final manuscript.
